RETRACTED

# Analysis of Prognostic Risk Factors of Sepsis Patients in Intensive Care Unit Based on Data Analysis

**DOI:** 10.1155/2022/3746640

**Published:** 2022-01-07

**Authors:** Lina Yao, Lei Zhang, Chengjie Zhou

**Affiliations:** Department of ICU, People's Hospital Affiliated to Ningbo University, Ningbo, Zhejiang, China

## Abstract

In this paper, a data-enabled analysis of the prognostic risk factors of sepsis patients in the intensive care unit is presented. For this purpose, we have selected 220 sepsis patients, preferably those admitted to the intensive care unit for treatment in a tertiary a hospital in Tianjin from June 2018 to June 2019 and received complete data as the research objects, to explore the prognostic risk factors of sepsis patients in the intensive care unit. All patients met the SSC sepsis diagnosis guidelines and recorded the patients' age, gender, underlying disease, and infection site. Laboratory indicators, such as blood routine, electrolytes, arterial blood gas, liver function, and renal function, were collected within 24 hours of admission. Furthermore, the corresponding specimens were cultured for pathogenic microorganisms according to the site of infection. The LAC value was measured at admission and 24 h after admission, and the 24 h lactate clearance rate was calculated. The Acute Physiological and Chronic Health Status Score II (APACHE-II) and SOFA score were calculated, which were based on the worst value of the index within 24 hours after admission. According to the prognosis of patients during hospitalization, they are divided into two groups: (i) survival group and (ii) death group. We entered all the data into Excel and used SPSS21.0 statistical software for data analysis and processing. Quantitative data are tested for normality. Quantitative data for normal distribution are expressed as mean ± standard deviation, and normal distribution and uniform variance are measured. The factors affecting the prognosis of patients with sepsis were first subjected to a single-factor logistic regression analysis, and a multiple logistic regression analysis was performed on the basis of the significance of the single-factor analysis. The results found that the prognosis of patients with sepsis in the ICU is affected by multiple factors such as underlying diseases, infectious microorganisms, comorbidities, and interventional therapy. APACHE-II score, 24 h lactate clearance rate, ARDS, and DIC are independent risk factors that affect the prognosis of ICU patients.

## 1. Introduction

Sepsis is a systemic inflammatory response syndrome (SIRS) caused by the presence of various pathogenic microorganisms and their toxins in the blood or tissues. It is generally caused by trauma, burns, shock, infection, and surgical operations and other clinically critical diseases. Those with more severe illness can progress to severe sepsis, septic shock, and multiple organ dysfunction syndrome, which is clinically one of the main causes of death in critically ill patients. It is common in complications caused by major surgery, severe infection, shock, and severe trauma. Clinical studies have shown that pathogenic bacteria invade the body to destroy the normal balance of anti-inflammatory and proinflammatory reactions in the body, which is the pathogenesis of sepsis. Related investigations and studies have shown that sepsis has a higher morbidity and fatality rate in ICU. In recent years, with the increase of invasive operations, the number of patients has increased, and the fatality rate has exceeded 50%. This has become a major problem that the current ICU treatment needs to face and poses a great threat to human health. Sepsis is divided into three types: sepsis, severe sepsis, and septic shock. At present, the fatality rates of domestic sepsis, severe sepsis, and septic shock have reached 13.82%, 35.43%, and 52.65% respectively. The severe situation cannot be ignored and can be described as another important research topic in clinical medicine [1–5].

RETRACTED

In view of the high morbidity and fatality rate of sepsis disease itself, it is very important to make prognostic analysis and research on it. Throughout the various clinical studies and publications that have appeared and implemented in the medical field, there are relatively few studies on the prognostic factors of sepsis. The number of cases in the existing studies is small, and it is a univariate analysis. There is no clear explanation for the prognostic interference factors. The specific influencing factors are not clear, and the analyzed factors themselves have certain limitations. Therefore, the analysis and research on the factors affecting the prognosis of sepsis has certain practical significance and practical value and can effectively fill a gap in the prognosis research of the disease in medicine. In foreign clinical studies of sepsis, it is pointed out that the case-fatality rate of patients with this type of disease will increase with the duration of the disease and the length of admission to the hospital. Once the best treatment period is missed, and no timely intervention is performed, sepsis will further increase. It develops and worsens and eventually evolves into MODS and septic shock, which increases the mortality rate. Another study by foreign scholars has shown that, in the group of patients with sepsis, elderly people over 60 years old account for a large proportion, reaching 65.2%. At the same time, as the age increases, the fatality rate of sepsis also increases. It suggests that age may be one of the prognostic factors. As sepsis has gradually become an important difficulty and subject content in clinical medical research, clinical research on sepsis has also begun to increase, and many clinical treatment results have been obtained, and valuable diagnosis and treatment experience has been accumulated. Comprehensive progress and updates have also been made in terms of the definition of the nature of the disease, diagnosis and treatment, and treatment standards of sepsis [6–10].

RETRACTED

Pathogenesis of sepsis is more complicated, prognostic factors have not made substantial progress, and there is a lack of valuable research and scientific and accurate conclusions. Therefore, it has become an important reason for the high fatality rate of sepsis caused by delayed intervention and treatment, so it is necessary to analyze and study the prognostic factors of sepsis. Not only can it enhance the cognition and mastery of sepsis between doctors and patients but can also help doctors to effectively intervene and observe the development and changes of sepsis patients and then make reasonable judgments and correct diagnosis and treatment, in order to achieve the purpose of improving the clinical treatment effect of sepsis and reducing the mortality rate.

Based on a retrospective research method, in this article, we have selected 220 sepsis patients with complete data who were treated in the ICU ward of a third-class hospital in Tianjin, particularly from June 2018 to June 2019, as the research object. All patients met the diagnostic criteria for sepsis. By analyzing the results of related laboratory examinations and the prognosis of patients, the relevant factors affecting the prognosis of patients with sepsis are explored, so as to provide a basis for effective treatment of the disease in clinical and the reduction of the mortality rate in the hospital.

The remaining portions of these articles are organized as follows: in the subsequent section, a brief, but thorough, review of the existing literature is presented, where the focus is on the sepsis related diseases. In Section 3, the proposed mechanism is presented, where sophisticated detail is provided about various parts of the proposed setup. Experimental results and observations were presented in Section 4. Finally, concluding remarks and future directives are provided in the last section.

## 2. Related Work

The concept of sepsis was first proposed in 1991 by the American College of Chest Physicians and the Society of Critical Care Medicine, which strengthened the understanding of the disease. In 2001, the American Academy of Critical Care Medicine and other institutions revised the criteria for sepsis, and indicators related to inflammation entered the diagnostic criteria for the disease, deepening the understanding from the perspective of the etiology. A year later in Spain, ESICM/SCCM/ISF published the famous Barcelona Declaration on Sepsis at the European Critical Care Medicine Conference [11, 12].

RETRACTED

Studies have shown that when a patient's infection is severe, systemic inflammation is formed in the body, which usually activates the anticoagulant system and coagulation system in the body, and inhibits the fibrinolytic system, leading to coagulation dysfunction. Once the coagulation system is activated, the concentration of anticoagulation factor proteins S, C, and antithrombin in the plasma decreases, and the concentration levels of TATC, prothrombin fragment *F*1 + 2, and soluble tissue factor are increased. Toxic disease progresses, coagulation factors are consumed, and APTT and PT are prolonged. The activation of the fibrinolytic system increased the levels of PAI-1, PAPC, D-dimer, and tissue-type plasminogen activator. Stimulating the procoagulant system usually leads to an increase in mortality. A large number of studies have shown that coagulation function can be stimulated by inflammatory response, and the activity of inflammatory response is affected by coagulation function. The two are highly correlated. Due to the procoagulant state formed by inflammation, inflammatory factors such as TNF-*α*, IL-1, and IL-6 participate in the formation of blood vessel thrombus and DIC in the body, which directly lead to serious damage to the body of patients with sepsis [13–18].

Studies have found that, after the initial explosive inflammatory response, an anti-inflammatory response is gradually induced, causing the patient to cause a secondary infection or the treatment is ineffective and fails. The apoptosis of epithelial cells, lymphocytes, and dendritic cells causes compensatory anti-inflammatory reactions such as decreased Th1 cell proliferation, low T lymphocyte reactivity, and ineffective antigen presentation, which is also called immune paralysis. Immune cell apoptosis is related to the host response caused by a variety of bacteria and many apoptotic pathways and has a very complex production mechanism [19–22].

The literature mentioned [23] to detect the blood lactic acid level of 50 patients with sepsis. The change curve of blood lactate over time was recorded, and the correlation between the prognosis of sepsis and blood lactate level was discussed. Through discussion, the author believes that increased blood lactic acid levels reduce the survival rate of patients with sepsis. Reducing the blood lactic acid concentration of patients with sepsis can improve the survival rate of patients. Finally, it is concluded that the survival rate of patients with sepsis is closely related to the blood lactic acid level of the body. The literature analyzed the value of lactic acid clearance rate on the clinical prognosis of patients with severe sepsis. It is pointed out that the blood lactate clearance rate can reflect the severity and prognosis of patients with severe sepsis. The lower the blood lactate clearance rate, the more severe the disease and the worse the prognosis [24]. The literature has studied the prognostic factors of 55 patients with sepsis. Through observation results pointed out that patients with sepsis PLT decreased, APTT time prolonged and INR increased, serum ALB level decreased, and APACHE-II score of more than 25 points all indicate worsening of the disease and poor prognosis [25].

RETRACTED

## 3. Materials and Methods

### 3.1. Research Object and Group

In this study, 220 patients with sepsis, who were admitted to the intensive care unit for treatment in a tertiary A hospital in Tianjin from June 2018 to June 2019 with complete data, were used as clinical research subjects, including 147 males and 73 females. According to the prognosis of patients during hospitalization, they were divided into survival group and death group. There were 101 patients in the death group and 119 patients in the survival group. Among them, there were 69 males in the death group and 32 females, aged 26–79 years. The average age was 63.1 ± 1.6 years. There were 78 males and 41 females in the survival group, aged from 27 to 79 years, with an average age of 61.2 ± 1.6 years.

### 3.2. Clinical Diagnostic Criteria

The diagnostic criteria included a clear or suspected infection, accompanied by some of the following general indicators: fever (body temperature>38.3°C); hypothermia (central body temperature <36.0°C); heart rate>90 beats/min or greater than 2 standard deviations of the normal heart rate range of different ages; shortness of breath, breathing rate>30 beats/min; changes in consciousness; obvious edema or positive fluid balance (>20 mg/kg over 24 hours); hyperglycemia (blood sugar>140 mg/dL or 7.7 mmol/L) without history of diabetes.

Inflammatory response parameters included leukocytosis (white blood cell count>12 × 109/L); leukopenia (white blood cell count<4 × 109/L). The white blood cell count is normal, but the immature white blood cell is > 0.10. Plasma C-reactive protein was > 2 standard deviations from the normal value. Precalcitonin was > 2 standard deviations from the normal value.

RETRACTED

Hemodynamic parameters included hypotension (systolic blood pressure <90 mmHg, mean arterial pressure <70 mmHg, or adult systolic blood pressure drop >40 mmHg, or drop by age >2 standard deviations); mixed venous blood oxygen saturation >0.70; cardiac bleeding index >58.3 ml/s·m.

Organ dysfunction parameters included hypoxemia (oxygenation index PaO2/FiO2<300 mmHg); acute oliguria (urine volume <0.5 ml/kg·h or osmotic concentration of 45 mmol/L for at least 2 h); creatinine increased ≥4.4 mmol/L; abnormal coagulation (international normalized ratio >1.5 or partially activated thromboplastin time >60 s); abdominal distension (bowel sounds disappear); thrombocytopenia (PLT < 100 × 109/L); hyperbilirubinemia (TBIL > 7.0 mmol/L).

Tissue perfusion parameters included hyperlactic acidemia (>1 mmol/L). The capillary refilling time is prolonged or the skin appears mottling.

### 3.3. Inclusion and Exclusion Criteria

This study included the following eligible patients: patients who were diagnosed with sepsis based on clinical symptoms and signs, laboratory examination results, and so on and were hospitalized in the intensive care unit of our hospital; being over 18 years old and under 80 years old. The hospitalization time was more than 24 hours, and the data of the included subjects were complete.

Those with the following conditions are excluded: age <18 years old or age >80 years old; definite diagnosis of primary or secondary adrenal insufficiency; patients with immune diseases who have been treated with glucocorticoids in the past year; patients who have used glucocorticoids in the past two weeks. Human immunodeficiency virus (HIV) positive is test during pregnancy and breastfeeding.

### 3.4. Research Method

Using the method of retrospective investigation and analysis, 220 sepsis patients with complete data who were treated in the ICU ward of a tertiary hospital from June 2018 to June 2019 were selected as the clinical research objects. According to the patient's prognosis, all sepsis patients are divided into two groups: survival group and death group, and the patient's age, gender, vital signs at the time of admission, infection site, underlying disease were recorded. Laboratory indicators, such as blood routine, electrolytes, arterial blood gas, liver function, and renal function, were collected within 24 hours of admission, and corresponding specimens were cultured for pathogenic microorganisms according to the site of infection. The LAC value was measured at admission and 24 h after admission, and the 24 h lactate clearance rate was calculated. The Acute Physiological and Chronic Health Status Score II (APACHE-II) and SOFA score were calculated based on the worst value of the indicators within 24 hours after admission. And the patient's organ function is good, whether there is failure and septic shock, and the relevant diagnosis and treatment measures are taken. A series of biochemical indicators are checked and measured for patients, including oxygenation index, blood lactate (Lac), 24 h lactate clearance, serum procalcitonin (PCT), C-reactive protein (CRP), total bilirubin (TBiL), platelet count (PLT), clotting time (PT), albumin (ALB), urea nitrogen (BUN), white blood cell count (WBC), aspartate aminotransferase (AST), alanine aminotransferase (ALT), creatinine (Cr) and creatine kinase isoenzyme (CK-MB), and many other project parameter indicators.

RETRACTED

### 3.5. Statistical Method

We have used Excel to build a database for all basic patient data. In this study, SPSS21.0 statistical software was used to perform statistical analysis and processing on all research test data, and the results of all measurement data were expressed in the form of mean ± standard deviation. The two groups of patients were compared and analyzed by independent sample *t*-test, and all count data were measured and compared with each index using the *x*^2^ test. According to the patient's survival or death, a single-factor analysis was performed, and statistically significant indicators were obtained for the study of the method of multiple logistic regression analysis.

## 4. Experimental Results

### 4.1. General Data Research and Analysis

Among the 220 patients in this clinical investigation, there are 147 males and 73 females. There are 101 patients in the death group and 119 patients in the survival group. Among them, there are 69 males in the death group and 32 females, aged 26∼79 years, with an average age of 63.1 ± 1.6 years. In the surviving group, there were 78 males and 41 females, aged 27–79 years, with an average age of 61.2 ± 1.6 years. There was no statistical difference between the death group and the survival group in terms of gender, average age, and age <60 years. The proportion of the death group ≥60 years old was more than that of the survival group. The proportion of people in the death group in terms of Gram-negative bacterial infection, fungal infection, combined ARDS/AKI/DIC, and the number of failed organs was higher than that in the survival group. The proportion of Gram-positive bacterial infection was lower than that of the survival group, and the difference was statistically significant. There was no difference in the proportion of infection sites, myocardial injury, septic encephalopathy, acute liver injury, and stress ulcer. The proportion of patients with cardiac insufficiency in the death group was higher than that in the survival group. There was no difference between the two groups in the proportion of people suffering from diabetes, COPD, and hypertension, and the difference was not statistically significant. The proportion of the survival group receiving anticoagulation therapy and continuous blood purification was higher than that of the death group. There was no difference in the time of receiving TPN treatment and mechanical ventilation between the two groups. There was no difference in the length of hospitalization between the survival group and the death group, and the difference was not statistically significant (Table 1 for details). GNI is Gram-negative infection. GPI is Gram-positive infection. FI is fungal infection. MI is myocardial injury. SE is septic encephalopathy. ALI is acute liver injury. SU is stress ulcer. AT is anticoagulant therapy. MVT is mechanical ventilation time. CBP is continuous blood purification.

RETRACTED

### 4.2. Clinical Laboratory Index Comparison

Comparing the survival group and the death group, there was no difference between the two in WBC, TBiL, PLT, oxygenation index, ALT, CK-MB, Cr, BUN, AST, ALB, PT, and PH, and there was no statistical significance. There were differences between the two groups in Lac, 24 h lactate clearance, CRP, PCT, APACHE-II scores, and SOFA scores, and the differences were statistically significant. The Lac, APACHE-II, and SOFA scores of the death group were higher than those of the survival group, and the 24-h lactate clearance rate was lower than that of the survival group (Table 2 and Figure 1). OI is the oxygen index. LACR is lactic acid clearance rate.

### 4.3. Logistic Analysis of Single Factors Affecting the Prognosis

A univariate analysis of influencing factors that may affect the prognosis of patients during hospitalization was carried out. The results showed that age, PCT, Lac, SOFA score, APACHE II score, 24 h lactic acid clearance rate, fungal infection, Gram-negative bacterial infection, comorbidities, receiving anticoagulation therapy, and continuous blood purification are the prognostic factors of patients (Table 3).

### 4.4. Multivariate Logistic Analysis Affecting the Prognosis

The method of multiple logistic regression analysis was used to perform multiple logistic regression with meaningful indicators obtained by univariate analysis as independent variables. The results showed that APACHE-II score, 24 h lactate clearance rate, ARDS, and DIC are independent risk factors affecting the prognosis of patients with sepsis (Table 4).

## 5. Discussion

Among 220 ICU patients with sepsis in this clinical investigation and study, there were 101 deaths and case-fatality rate of 45.91%. Through performing a retrospective analysis of their clinical cases, the aim is to explore the prognosis of patients with sepsis and the factors in order to provide more theoretical basis and help in the clinical prevention and treatment of sepsis. Through this analysis and research, the factors affecting the prognosis of patients with sepsis in the ICU are concluded, which may include age, PCT, Lac, SOFA score, APACHE-II score, 24 h lactic acid clearance rate, combined fungal infection, Gram-negative bacterial infection, combined AKI/ARDS/DIC, receiving anticoagulation therapy, continuous blood purification, and others. The multivariate logistic regression analysis showed that the independent factors affecting the prognosis of patients may be APACHE-II score, 24-hour lactate clearance rate, combined ARDS, and combined DIC.

RETRACTED

From the research of this clinical investigation, it is not difficult to see that the mortality rate of sepsis patients aged ≥60 years is high, while the mortality rate of sepsis patients aged <60 years is low, and there is a statistical difference. It can be considered that an age ≥60 years may be a risk factor affecting the prognosis of ICU patients with sepsis, but multivariate logistic regression analysis shows that an age ≥60 yearsis not an independent risk factor affecting the prognosis of ICU patients with sepsis.

It is not difficult to see from this clinical study that the prognosis of sepsis is judged by a single-factor analysis. APACHE-II score ≥20 points is a risk factor that affects the prognosis of patients. Among them, sepsis patients with APACHE-II score ≥20 points have a high mortality rate, and sepsis patients with APACHE-II score <20 points have a low mortality rate. Obviously from the data results, the fatality rate of sepsis patients with APACHE-II score ≥20 points is much higher than that of patients with APACHE-II score <20 points. Multivariate logistic regression analysis found that APACHE-II score ≥20 points is an independent risk factor for death in patients with sepsis.

Through the analysis of various markers of sepsis, it is found that PCT is not only meaningful for assessing the prognosis of patients but is also an indicator for judging the severity of the patient's infection. Moreover, PCT is not affected by the immune suppression state of the body. The degree is generally related to the severity of the infection. In this study, the PCT level of patients in the death group was higher than that in the survival group, and single-factor logistic regression analysis found that PCT was a risk factor for the prognosis of patients.

RETRACTED

This study found that the death group was compared with the survival group. The lactate of the death group was significantly higher than that of the survival group, and the 24-hour lactate clearance rate of the death group was significantly lower than that of the survival group. The comparison between the two was statistically significant. Considering that the 24-hour lactate clearance rate may be an independent factor affecting the prognosis of patients with sepsis. Therefore, dynamic monitoring of blood lactic acid value during the patient's ICU hospitalization, timely active fluid resuscitation, improvement of tissue perfusion, and control of lactic acid level may be an effective way to improve the prognosis of the population and extend the survival time.

According to this investigation and research, single-factor and multifactor analysis of the factors affecting the prognosis of sepsis were conducted. Combined fungal infections are closely related to the prognosis of patients with sepsis. For patients with sepsis, especially severe sepsis, invasive auxiliary support and high-dose broad-spectrum antibiotics are mainly used to treat patients with organ functions. In normal operation, it is very easy to cause an imbalance in the flora of the patient's body, causing the body's immune protection function to be destroyed and the chance of the body to be infected with fungi increases, making the disease worse and accelerating the death of the patient. Therefore, it is not difficult to find the important influence of fungal infection factors on the prognosis of patients with sepsis.

In this clinical investigation and study, in terms of the fatality rate of patients with sepsis combined with AKI, the death group was obviously higher than that of the survival group. A univariate analysis showed that sepsis combined with AKI is a risk factor affecting the prognosis of patients, one of the important reasons for the increased mortality of patients with sepsis. Therefore, effective prevention and treatment of sepsis combined with AKI is a problem to be solved in critical care medicine.

From this clinical investigation and research, it is not difficult to see that, in terms of the mortality of patients with sepsis and ADRS, the death group is obviously higher than the survival group. Judging by univariate and multivariate prognostic analysis of sepsis, the prognostic factors of sepsis may include the factors of sepsis combined with ADRS. The fatality rate of patients with sepsis will increase significantly with the changes of sepsis with ADRS factors, which becomes one of the important causes of death in patients with sepsis.

In this study, the probability of DIC in the death group was significantly higher than that in the survival group, and it was statistically significant, indicating that DIC can aggravate the condition of sepsis and is an important factor in the high mortality rate. In the multiple logistic regression analysis, it is considered that sepsis complicated by DIC is a risk factor affecting the prognosis of patients. Sepsis complicated by DIC is an independent risk factor affecting the prognosis of patients with sepsis and early detection and improvement of coagulation dysfunction. Early and timely intervention may prevent the prognosis of sepsis and improve the survival rate of hospitalized patients with sepsis.

RETRACTED

When the inflammatory response is uncontrollable, the body will induce a violent response of inflammatory cells, a waterfall effect occurs, and the inflammatory response continues to expand. It can damage local tissues and a distant organ, and more severely, multiple organ dysfunction syndrome (MODS) may occur. This study found that the mortality rate of patients in the death group was higher than that of the survival group, which indirectly indicates that the number of organ failures is closely related to the mortality of patients.

From this clinical investigation and research, it is not difficult to see that the survival group is significantly larger than the death group, and the difference is statistically significant. Judging by single-factor and multifactor logistic regression scores, the use of anticoagulant therapy in the clinical treatment of ICU inpatients with sepsis can effectively reduce the mortality of patients. Anticoagulant therapy can be used as an influencing factor for the prognosis of sepsis.

In this study, the death group was compared with the survival group. The proportion of CBP treatment in the survival group was significantly higher than that of the death group. Unit logistic regression analysis, considering that continuous blood purification treatment is a protective factor for the prognosis of patients, proves that continuous blood purification can affect the prognosis of patients, indicating that continuous blood purification has a better effect on sepsis. Therefore, the prognosis of patients with sepsis may be better if CBP is added to intervention treatment on the basis of conventional treatment.

## 6. Conclusion

This study analyzed the single-factor logistic regression analysis to obtain age, PCT, Lac, SOFA score, APACHE-II score, 24 h lactic acid clearance rate, fungal infection, Gram-negative bacterial infection, comorbidities, receiving anticoagulation treatment rate, and continuity blood purification, which may be related to the prognosis of patients with sepsis in the ICU. Multivariate logistic regression analysis showed that APACHE-II score, 24 h lactate clearance rate, ARDS, and DIC are independent risk factors that affect the prognosis of ICU patients with sepsis.

RETRACTED

Regarding the research deficiencies and prospects, this research is a retrospective case analysis, with certain limitations. The number of cases included in the trial is small. If conditions permit, the number of cases from multiple hospitals can be collected. This article only collected the experimental data within 24 hours of the patient's admission and did not carry out continuous monitoring in the later stage. If you want to further study the changes in the patient's condition, further dynamic observations are needed. Therefore, for the analysis of factors affecting the prognosis of patients with sepsis in the intensive care unit, there are still not enough systematic and comprehensive deficiencies.

## Figures and Tables

**Figure 1:** Comparison of patient laboratory indicators.

**Table 1:** Comparative analysis of patients' general information.

Item		Group		*P*
		Survival group	Death group	
Gender	Male	78	69	0.138
	Female	41	32	0.130

Age	<60	50	26	0.158
	≥60	69	75	0.008

Site of infection	Lung	61	56	0.078
	Urinary	30	22	0.823
	Abdomen	13	14	0.245
	Others	15	9	0.151

Pathogen classification	GNI	43	89	0.005
	GPI	76	12	0.002
	FI	12	19	0.023

Organ disorders	ARDS	41	62	0.003
	AKI	34	67	0.000
	DIC	21	34	0.004
	MI	54	46	0.731
	SE	61	52	0.765
	ALI	27	23	0.265
	SU	66	57	0.481

Number of failed organs	1	91	34	0.005
	2	25	13	
	3	3	25	
	4	0	19	
	5	0	10	

Basic illness	Diabetes	23	24	0.356
	COPD	9	13	0.231
	Hypertension	53	45	0.981
	Heart failure	107	98	0.038

Treatment	TPN	81	57	0.168
	AT	77	48	0.027
	MVT	152.4	223.5	0.162
	CBP	38	13	0.008

Hospital stay	ICU time	12.6	9.6	0.276

**Table 2:** Comparison of patient laboratory indicators.

Index	*P*	Index	*P*	Index	*P*
WBC	0.08	Lac	0.02	BUN	0.53
TBil	0.57	PH	0.16	AST	0.08
PLT	0.39	LACR	0.02	ALB	0.08
PCT	0.00	ALT	0.09	PT	0.47
CRP	0.00	CK-MB	0.28	APACHE II	0.00
OI	0.19	Cr	0.78	SOFA	0.00

**Table 3:** Single-factor analysis of prognostic factors.

Item	*β*	SE	Wals	df	Sig	OR	95% CI
Age	0.16	0.76	2.61	1	0.008	1.09	1.06
PCT	0.22	0.08	7.28	1	0.004	1.24	1.05
Lac	0.29	0.13	4.88	1	0.025	1.34	1.25
SOFA	0.70	0.57	1.91	1	0.034	2.07	1.97
APACHE	5.66	0.67	6.55	1	0.015	2.46	2.35
LACR	−7.31	0.54	1.66	1	0.005	0.16	0.000
FI	1.14	0.58	0.56	1	0.017	0.56	1.49
GNI	1.11	0.53	1.46	1	0.003	1.98	1.88
DIC	0.96	0.37	6.85	1	0.013	5.16	2.84
ARDS	1.25	0.45	17.65	1	0.000	2.55	1.48
AKI	0.53	0.44	1.46	1	0.014	1.35	1.26
AT	-1.25	0.41	11.26	1	0.002	0.54	0.34
CBP	−1.41	0.46	8.92	1	0.002	0.97	0.92

RETRACTED

**Table 4:** Multivariate logistic analysis affecting prognosis.

Item	*β*	SE	Wals	df	Sig	OR	95% CI
APACHE	0.83	0.38	4.79	1	0.027	2.29	1.09
LACR	−7.29	0.43	6.01	1	0.024	0.00	0.00
ARDS	1.24	0.35	12.06	1	0.003	3.48	1.68
DIC	1.59	0.64	6.13	1	0.015	4.92	1.39

## Data Availability

The datasets used are available from the corresponding author on reasonable request.
